The article "Xiao-Qing-Long-Tang shows preventive effect of asthma in an allergic asthma mouse model through neurotrophin regulation" was published in 2013. Journal: BMC Complement Altern Med.

# Xiao-Qing-Long-Tang shows preventive effect of asthma in an allergic asthma mouse model through neurotrophin regulation

**DOI:** 10.1186/1472-6882-13-220

**Published:** 2013-09-08

**Authors:** Ren-Shiu Chang, Shulhn-Der Wang, Yu-Chin Wang, Li-Jen Lin, Shung-Te Kao, Jiu-Yao Wang

**Affiliations:** 1 Graduate Institute of Chinese Medicine, China Medical University, No. 91 Hsueh-Shih Road, Taichung, 40402, Taiwan; 2 School of Post-Baccalaureate Chinese Medicine, College of Chinese Medicine, China Medical University, No. 91 Hsueh-Shih Road, Taichung 40402, Taiwan; 3 School of Chinese Medicine, College of Chinese Medicine, China Medical University, No. 91 Hsueh-Shih Road, Taichung 40402, Taiwan; 4 Department of Chinese Medicine, China Medical University Hospital, No. 2 Yude Road, Taichung, 40447, Taiwan; 5 Department of Pediatrics, College of Medicine, National Cheng Kung University, No. 138, Sheng-Li Road, Tainan 70428, Taiwan; 6 Department of Chinese Medicine, Tainan Sin-Lau Hospital, No. 57, Sec. 1, Dongmen Rd, Tainan 70142, Taiwan

**Keywords:** Asthma, Xiao-Qing-Long-Tang (XQLT), Nerve growth factor (NGF), Brain-derived neurotrophic factor (BDNF), p75 neurotrophin receptor (p75NTR)

## Abstract

**Background:**

This study investigates the effect of Xiao-Qing-Long-Tang (XQLT) on neurotrophin in an established mouse model of Dermatophagoides pteronyssinus (Der p)-induced acute allergic asthma and in a LA4 cell line model of lung adenoma. The effects of XQLT on the regulation of nerve growth factor (NGF) and brain-derived neurotrophic factor (BDNF), airway hyper-responsiveness (AHR) and immunoglobulin E were measured.

**Methods:**

LA4 cells were stimulated with 100 μg/ml Der p 24 h and the supernatant was collected for ELISA analysis. Der p-stimulated LA4 cells with either XQLT pre-treatment or XQLT co-treatment were used to evaluate the XQLT effect on neurotrophin.

Balb/c mice were sensitized on days 0 and 7 with a base-tail injection of 50 μg Dermatophagoides pteronyssinus (Der p) that was emulsified in 50 μl incomplete Freund’s adjuvant (IFA). On day 14, mice received an intra-tracheal challenge of 50 μl Der p (2 mg/ml). XQLT (1g/Kg) was administered orally to mice either on days 2, 4, 6, 8, 10 and 12 as a preventive strategy or on day 15 as a therapeutic strategy.

**Results:**

XQLT inhibited expression of those NGF, BDNF and thymus-and activation-regulated cytokine (TARC) in LA4 cells that were subjected to a Der p allergen. Both preventive and therapeutic treatments with XQLT in mice reduced AHR. Preventive treatment with XQLT markedly decreased NGF in broncho-alveolar lavage fluids (BALF) and BDNF in serum, whereas therapeutic treatment reduced only serum BDNF level. The reduced NGF levels corresponded to a decrease in AHR by XQLT treatment. Reduced BALF NGF and TARC and serum BDNF levels may have been responsible for decreased eosinophil infiltration into lung tissue. Immunohistochemistry showed that p75NTR and TrkA levels were reduced in the lungs of mice under both XQLT treatment protocols, and this reduction may have been correlated with the prevention of the asthmatic reaction by XQLT.

The article "Xiao-Qing-Long-Tang shows preventive effect of asthma in an allergic asthma mouse model through neurotrophin regulation" was published in 2013. Journal: BMC Complement Altern Med.

**Conclusion:**

XQLT alleviated allergic inflammation including AHR, IgE elevation and eosinophil infiltration in Der p stimulated mice by regulating neurotrophin and reducing TARC. These results revealed the potential pharmacological targets on which the XQLT decotion exerts preventive and therapeutic effects in an allergic asthma mouse model.

## Background

The pathology of allergic asthma is characterized by clear eosinophil infiltration in the airways and the elevation of systemic IgE levels, mediated by type 2 T-helper (Th2) cells and cytokines. Airway remodeling, observed in severe form of allergic asthma, is a consequence of repetitive airway inflammation and Th2-type reaction. Although the imbalance of Th1/Th2 immune response is well known and has been used to elucidate the immune-pathogenesis of allergy and other autoimmune diseases, this relevant theory is incomprehensive and satisfactory clinical applications are lacking. Traditional Chinese Medicine (TCM) decotion such as Xiao-Qing-Long-Tang (XQLT) is frequently used in Asia for the clinical treatment of bronchial asthma and allergic rhinitis [1,2], XQLT, in particular, has been found to have beneficial effects in relieving Th2-based reactions in the airways of animal models of allergic asthma [3-6]. Despite its effects on immunological regulation, the molecular mechanism and pharmacological action of XQLT remain unclear. XQLT is highly popular in TCM and complementary medicine, because it has no major side effects. Therefore, the therapeutic targets and ethno-pharmacological action of the decotion must be thoroughly examined before it can be widely used for the prevention and treatment of asthma.

Members of the neurotrophin family have been shown not only to act as growth factors in the nervous system, but also to act as pro-inflammatory factors in the immune system. Airway hyper-responsiveness (AHR) can be mediated through substance P, neurokinin A, and other members of the neurotrophin family, suggesting that neural hyper-innervation of the airways may be responsible for AHR [7]. Nerve growth factor (NGF) which is a member of the neurotrophin family is one product of activated Th2 cells [8,9]. Moreover, our recent research demonstrated that a major allergen of house dust mite, *Dermatophagoides pteronyssinus* Group 2 (Der p 2) could induce NGF production and reactive oxygen species in the airway, as well as allergic inflammation after direct intra-tracheal instillation into the lungs of mice [10].

The article "Xiao-Qing-Long-Tang shows preventive effect of asthma in an allergic asthma mouse model through neurotrophin regulation" was published in 2013. Journal: BMC Complement Altern Med.

NGF and the brain-derived neurotrophic factor (BDNF) are survival and activation factors of eosinophil in patients with allergic bronchial asthma [11]. NGF and BDNF are expressed in multiple cells, including epithelial cells, active immune cells, and neural cells. In allergic asthma, the tissue that is primarily responsible for allergen presentation is the bronchiolar epithelium. These epithelial cells present allergens and induce allergy pathways that involve multiple events, including dendritic cell activation and chemokine secretion [12,13]. Moreover, NGF and BDNF have been observed at elevated concentration in patients with allergic diseases. Although BDNF has not yet been implicated in early allergic reactions as NGF, its role in allergic airway dysfunction has been found to be important [14]. BDNF is now known to be directly involved in airway smooth muscle hyperplasia and hypertrophy by interacting with tyrosine kinase B (TrkB), but not with p75 neurotrophin receptor (p75NTR), and through the secretion of metalloproteinase-9 (MMP-9) [15,16]. BDNF is also known responsible for neuronal plasticity in brain and lung. Neuronal plasticity is also a key factor in airway remodeling and airway hyper-responsiveness. p75NTR is required for BDNF in regulating depression or anxiety in brain function, but it is not a necessary factor in smooth muscle hypertrophy which result in airway remodeling [17,18]. p75NTR is a low-affinity receptor of all factors of the neurotrophin family, and allergic inflammation and eosinophil infiltration have been eliminated in p75NTR-knockout mice [19,20]. p75NTR is known for inducing NF-κB activation that has been demonstrated to be a major transcriptional factor in the Th2-type immune response [21,22]. NGF may also affect dendritic cells (DCs) through p75NTR [23].

This paper presents our findings that XQLT inhibited the production of the members of the neurotrophin family in a mouse model of allergic asthma, alleviating AHR and the allergic inflammation of the airway. LA4 is a bronchial epithelial cell line of murine lung origin and produces NGF in response to Der p allergen [10]. XQLT has been found to inhibit NGF and BDNF and p75NTR expression in LA4 cells. These results identified the potential pharmacological targets of the XQLT decotion that might exert its preventive and therapeutic effects in a mouse model of allergic asthma.

## Methods

### TCM preparation: Xiao-Qing-Long-Tang (XQLT)

XQLT extract powder was kindly provided by KO-DA Pharmaceutical Co. (Taoyuan, Taiwan, R.O.C.). All of the eight herbs listed in description below were originally grown in mainland China and collected by the KO-DA Pharmaceutical Co. from professional herbal growers. The voucher specimens have been deposited in the publicly available herbarium of KO-DA Pharmaceutical Co. Those eight herbs were authenticated by Professor Shih-Chang Lee, China Medical University, Taiwan. The XQLT extract was prepared as described in a previous study [24]. Briefly, eight herbal ingredients were mixed by proportion which is shown as number that is in the brackets behind each scientific name of herbal. They were *Pinellaiae tuber* (6.0, root of *Pineliaternata breitenbach*), *Ephedrae herba* (3.0, stem of *Ephedra sinica Stapf*), *Schizandrae fructus* (3.0, a fruit of *Schizandra chinensis Baill.*), *Cinnamonomi cortex* (3.0, cortex of *Cinnamomum cassia Blume*), *Paeoniae radix* (3.0, root of *Paeonia lactiora Pall.*), *Asariherba cum radice* (3.0, whole plant of *Asiasarum heterotropoides F. Maekawa var. mandshuricum F. Maekawa*), *Glycyrrhizae radix* (2.0, root of *Glycyrrhiza uralensis Fisch. Et. DC*), and *Zingiberis siccatum rhizoma* (1.0, steamed root of *Zingiber officinale Roscoe*). The mixture was extracted sequentially with 17.5 L and 12.5 L boiling water each time for 1 h. The extracted liquid was mixed and filtered. After filtration, the dregs of the decotion were removed. The filtered liquid was lyophilized then crushed into a thin powder. The yield of dried extract from starting crude material was 661.8 g (26.4%, w/w). The dried extract was subsequently used for all experiments in this research. The batch number of XQLT extract is 98041021.

The article "Xiao-Qing-Long-Tang shows preventive effect of asthma in an allergic asthma mouse model through neurotrophin regulation" was published in 2013. Journal: BMC Complement Altern Med.

The XQLT mixture was suspended in distilled water to a fixed concentration for being orally administered to the mice through feeding needle and swallowing. The feeding volume was adjusted within 0.2~0.3 ml to avoid mice of pain. For *in vitro* use, the XQLT mixture was dissolved in distilled water, after which the solution was centrifuged at 7500 rpm for 30 min. Following filtration, the aqueous extract was lyophilized and weighed. This XQLT extract was re-dissolved in pyrogen-free isotonic saline (YF Chemical, Taipei, Taiwan) and filtered through a 0.22-μm filter (Microgen, Laguna Hills, CA, USA). A sample of the filtered pyrogen-free solution was lyophilized and weighed. The final concentration of the last filtered pyrogen-free solution was estimated by the sample. The filtered pyrogen-free solution was stored at -20°C until use.

### Production of neurotrophin in cell lines following Der p stimulation

LA4 (murine lung adenoma) cell line was purchased from the Bioresource Collection and Research Center (BCRC, Hsinchu, Taiwan; BCRC60239 derived from ATCC: CCL-196). The LA4 cells were cultured in Ham’s F12 medium (Gibco), which contained 2.5 mM L-glutamine, 15% fetal bovine serum (FBS), and 0.1% gentamicin, in an incubator at 37°C with 5% CO_2_. Group XC comprised LA4 cells that were treated with XQLT alone for 24 h. Group XP comprised LA4 cells that were treated with XQLT for 1 h, then the XQLT was washed out, subsequent to 24 h Der p stimulation. Group XD comprised LA4 cells which were simultaneously treated with XQLT and Der p for 24 h. Group D comprised LA4 cells which were treated with Der p alone for 24 h. Group N comprised entirely untreated LA4 cells. 1 mg/ml XQLT and 100 μg/ml Der p concentrations set following a pre-titration trial (data not shown) were administered to the cells in all groups. After the treatment of all cell groups for 24 h, supernatants and total cell protein were collected for analysis. All the protocols were schematic in Figure 1A. LA4 cells were all seeded at concentration of 1×10^6^ cells/ ml.

**Figure 1:** **XQLT inhibited NGF, BDNF, TARC and p75NTR expression in LA4 cells stimulated with Der p. Pre-treatment (XP) and co-treatment (XD) with XQLT in Der p-stimulated cells and merely XQLT treated cells (XC) were used to assess the effects of XQLT on neurotrophin and associated receptor. (A)** The supernatant was collected and analyzed by ELISA to obtain NGF, BDNF and TARC levels. Student’s t test was performed versus Group D. Schematic of cell experiment groups is also shown under those ELISA data. **(B)** Whole cell extracts were used for western blotting with anti-p75NTR antibody or anti-NGF antibody (commercial antibody also recognizes pro-NGF). Protein expression level was assessed as western band density detected by densitometry and was depicted as proportional bar plots (negative group level set as 1). Student’s t test was performed versus Group D. All the experiments in **(A)** and **(B)** were repeated for at least three times. The values shown are means ± SD. * means p < 0.05, ** means p < 0.01, *** means p < 0.005 in **(A)** and **(B)**.

### Western blot analysis of NGF and p75NTR expression in cell lines

Cells (1~2 × 10^6^ cells/ml) were lysed using a Triton X-100-based lysis buffer that contained 1% Triton X-100, 150 mM NaCl, 10 mM Tris (pH 7.5), 5 mM EDTA, 5 mM NaN_3_, 10 mM NaF, and 10 mM sodium pyrophosphate. Cell extracts were separated using SDS-PAGE, then transferred to a PVDF membrane (Millipore Corporation, Billerica, MA, USA). After blocking, the blots were developed using rabbit polyclonal anti-p75NTR antibody or rabbit polyclonal anti-NGF antibody. The blots were then hybridized using HRP-conjugated goat anti-rabbit IgG (Calbiochem, San Diego, CA, USA) and developed with a chemiluminescence kit (Western Lightning Chemiluminescence Reagent PLUS; PerkinElmer Life Sciences Inc., Boston, MA, USA). The western band density that corresponded to the p75NTR or NGF or pro-NGF or β-actin was determined using an image analysis system. The detected density was representation of expression level of each protein. The density of p75NTR, NGF or pro-NGF was calculated versus density of β-actin and result was shown as proportion. The proportion was plotted as bar graph with the value of group N set to be 1. Single Antibody: anti-p75NTR {Abcam Inc. ab8874}; anti-NGF {NGF (M-20), SANTA CRUZ BIOTECHNOLOGY, INC. sc-549}.

The article "Xiao-Qing-Long-Tang shows preventive effect of asthma in an allergic asthma mouse model through neurotrophin regulation" was published in 2013. Journal: BMC Complement Altern Med.

### Acute asthma model set-up

Specific pathogen-free, 6~8 week-old female BALB/c mice from the Laboratory Animal Center of National Cheng Kung University were used in this study. The mice were housed in microisolator cages (Laboratory Products, Maywood, NJ, USA) and provided with sterile food and water *ad libitum*. All care and treatment of the experimental animals followed the guidelines set by the National Science Council of the Republic of China. The Institutional Animal Care and Use Committee (IACUC) of the China Medical University (Permit Number: 100-139-N) approved the protocol.

On days 0 and 7, groups of mice were subcutaneously injected at the base of their tails with a 50 μl emulsion that contained 50 μg of Der p in incomplete Freund’s adjuvant (IFA; Difco, Detroit, MI, USA). Fourteen days later, the mice were lightly anesthetized with an intra-peritoneal (i.p.) injection of 60 μg/kg body weight of sodium pentobarbital (Nembutal, Abbott Laboratories, North Chicago, IL, USA). The animals received intra-tracheal (i.t.) instillation with 50 μl of Der p (2 mg/ml) for the allergen challenge (AC), after which they were held in an upright position for 1 min, so that they could resume normal breathing. Figure 2A schematically depicts the complete protocol for XQLT treatment. The XQLT dose that was used in this study was based on the authors’ previous study [3] and the pilot study before this research. In Group D, the mouse model for an acute, Der p allergen-induced asthmatic attack was as follows: initial sensitization with Der p on Day 0, a Der p booster on Day 7, and an i.t. Der p AC on Day 14. The animals were sacrificed on Day 16. To evaluate the effects of XQLT on this model, mice in the therapeutic protocol (Group T) were given 1 g/kg BW of XQLT once at 24 h after AC, and mice in the preventive protocol (Group P) were given 1 g/kg BW of XQLT six times, every other day from Day 2 onward, with the last treatment administered 48 h before AC. Mice in Group XC (control) were administered 1 g/kg BW of XQLT every other day from Day 2 onward without Der p sensitization or AC. Group N (naive group) comprised animals without Der p sensitization, challenge or XQLT treatment. They were included in the experiments for comparison. Each group, associated with one experimental condition, comprised six mice.

The article "Xiao-Qing-Long-Tang shows preventive effect of asthma in an allergic asthma mouse model through neurotrophin regulation" was published in 2013. Journal: BMC Complement Altern Med.

**Figure 2:** **Respiratory flow resistance results showed inhibition of AHR by XQLT in a mouse model of Der p-induced acute asthma. (A)** Schematic of mice experiment groups. **(B)** Respiratory flow resistance was measured by intubation 2 d after Der p challenge. The standard curve chart displays resistance values under methacholine challenge ranging from 0 mg/ml to 4 mg/ml. Values represent the means ±SD (n = 6 mice for each group, all experiments repeated for at least three times). Student's t test was performed versus Group D (* means p < 0.01; ** means p < 0.005). Student’s t test was also performed between Group P and Group T (# means p < 0.05).

Lyophilized house dust mites (Dermatophagoides pteronyssinus; Der p) were purchased from Allergon (Engelholm, Sweden). Crude Der p preparation was extracted with ether. After dialysis with deionized water, the Der p extract was lyophilized and stored at -70°C until use. LPS concentration of the Der p preparations was 1.96EU/mg of Der p (Limulus amebocyte lysate test; E-Toxate; Sigma-Aldrich).

### Invasive measurement of airway resistance

The lung function of mice that had been anesthetized with sodium pentobarbital (60 μg/kg BW) was invasively analyzed. An 18-gauge stainless-steel cannula was inserted into the trachea of each mouse, which was placed on the FlexiVent system (Scireq^®^, Montreal, QC, Canada) for forced oscillation measurements after tracheostomy and consecutive examinations of total lung capacity (TLC). According to manufacturer’s instruction and previous studies [25,26], a single-compartment model of respiratory mechanics was used to evaluate lung function and the responses of the airway to methacholine (0 mg/ml to 4 mg/ml) 48 h after the Der p challenge. Total respiratory system resistance (Rrs) was measured using a snapshot perturbation maneuver. Methacholine was aerosolized for ventilation with an ultrasonic nebulizer for 10 s, and 12 snapshot perturbations were performed.

### Collection of serum and broncho-alveolar lavage fluid (BALF)

The following procedures were based on previous study [3,24] with slightly modification. The mice were sacrificed by administering a sodium pentobarbital overdose (20 mg/ml) following Der p challenge. After sacrifice, BALF was collected by flushing the lung with two separate normal saline through the trachea, around 1 ml of BALF was recovered. Cells were recovered from BALF by centrifugation at 200 × *g* for 5 min at 4°C, then washed in red blood cell lysis solution, and finally diluted with RPMI-1640 medium (GIBCO/BRL, Life Technologies, Inc., Gaithersburg, MD, USA). The total leukocyte content of the BALF was determined using a cytometer to be 1 × 10^5^ cells/ml. Blood was collected either through the axillary artery or directly from the heart. The collected blood was left to stand for 1 h at room temperature to clot. Centrifugation at 14,000 rpm removed the clotted matter to obtain the serum.

The article "Xiao-Qing-Long-Tang shows preventive effect of asthma in an allergic asthma mouse model through neurotrophin regulation" was published in 2013. Journal: BMC Complement Altern Med.

### Total and Der p-specific IgE/IgG1/IgG2a concentrations in the BALF and serum

IgE, IgG1, and IgG2a concentrations in the BALF and serum were measured using an ELISA kit (Bethyl Laboratories, Inc). The wells of a 96-well ELISA plate (Model No. 445101, NUNC) were coated with 100 μl of affinity-purified mouse antibody in 50 mM carbonate-bicarbonate buffer (pH 9.6). The plate was incubated at room temperature (20°C–25°C) for 1 h. After the antibody solution was removed, 200 μl of blocking solution that contained 50 mM Tris, 0.14 M NaCl, and 1% bovine serum albumin (BSA) (pH 8.0) was placed in each well and incubated at room temperature for 30 min. The plates were washed five times with PBST (0.05% Tween 20). The dilutions of BALF or serum with sample/conjugate diluent (50 mM Tris, 0.14 M NaCl, 1% BSA, 0.05% Tween 20) were added to the wells. After being sealed with adhesive tape, the plates were incubated at room temperature for 1 h and again washed five times. After 100 μl of diluted horseradish peroxidase (HRP)-conjugated antibody was added to each well, the plates were again incubated at room temperature (20°C–25°C) for 1 h. Thereafter, the plates were again washed five times, and 100 μl of tetramethylbenzidine (TMB) substrate solution was added to each well. The plates were then kept in the dark at room temperature for 15 min for fluorescence developing. The enzyme reaction was stopped by adding 100 μl of stop solution (0.18 M H_2_SO_4_). Absorbance was measured at a wavelength of 450 nm on an ELISA plate reader.

Antibody ELISA: Mouse IgE ELISA Quantitation Set, Bethyl Laboratories, Inc. E90-115; Mouse IgG1 ELISA Quantitation Set, Bethyl Laboratories, Inc. E90-105; Mouse IgG2 ELISA Quantitation Set, Bethyl Laboratories, Inc. E90-107;

### IFN-γ/ IL-5/IL-13/TGF-β1/TARC/NGF/BDNF concentrations in BALF, serum, and cell line supernatants

The concentrations of NGF and BDNF in the BALF, serum, and cell culture supernatant were measured using the appropriate ELISA kits (NGF & BDNF Emax Immuno-Assay Systems), according to the manufacturers’ instructions (Promega, Madison, WI, USA). The concentrations of IFN-γ, IL-5, TGF-β1, TARC and IL-13 in the BALF, serum, and cell culture supernatants were measured using an ELISA kit according to the manufacturer’s instructions.

The article "Xiao-Qing-Long-Tang shows preventive effect of asthma in an allergic asthma mouse model through neurotrophin regulation" was published in 2013. Journal: BMC Complement Altern Med.

Cytokine ELISA: NGF Emax^®^ ImmunoAssay System, Promega G7630; BDNF Emax^®^ ImmunoAssay System, Promega G7610; mouse IFN-gamma {R&D Systems, Inc. DuoSet ELISA DY485}; mouse IL-5 {R&D Systems, Inc. DuoSet ELISA DY405}; mouse TGF-beta1 {R&D Systems, Inc. DuoSet ELISA DY1679}; mouse IL-13 {R&D Systems, Inc. DuoSet ELISA DY413}.

### Lymphocyte/macrophage/neutrophil/eosinophil percentages in the BALF

BALF cells were spun down onto a glass slide at 360 rpm for 8 min by cytospinning. The slides were then dried and stained by the hematoxylin and eosin (H&E) or eosinophil-specific staining methods (Eosinophil-Mast Cell Stain Kit, CEM-1-IFU; ScyTek Laboratories, Inc., Utah, USA). More than 200 cells were counted under a photomicroscope and the percentages of lymphocytes, macrophages, neutrophils, and eosinophils were thereby determined.

### Immunohistochemistry

The entire lung was removed and embedded in paraffin for slicing. The paraffin lung slices were mounted on glass slides. The paraffin was then depleted at 60°C. Each slice was then sequentially treated with the following reagents; xylene, ethanol, 3% H_2_O_2_ (80% methanol) (v/v), and 0.01 M sodium citrate buffer (pH 6.0, 95°C). After 10% non-fat milk was used to block the cooled slice, a rabbit polyclonal anti-p75NTR antibody or a rabbit polyclonal anti-TrkA antibody (Abcam, Cambridge, UK) were used for immunostaining (4°C, overnight). Anti-Rabbit IgG antibody (FITC or Phycoerythrin conjugated; Abcam, Cambridge, UK) was used as a secondary antibody to develop fluorescence. The developed slice was observed under a light microscope. The area density of fluorescence was analyzed using an image analysis system. The fluorescence density results are shown as a bar graph. Single Antibody: anti-p75NTR {Abcam Inc. ab8874}; anti-TrkA antibodies {Abcam Inc. ab76291}.

### Statistical analysis

The data are presented as mean ± standard deviation. Statistical comparisons were performed using Student’s t test analysis, with significance set at P < 0.05 or as indicated in each figure legend (two-sided test). All the statistical differences are indicated in the figure legends.

## Results

### XQLT inhibited NGF, BDNF, and p75NTR expression in LA4 cell line following Der p stimulation

An *in vitro* model of mouse lung adenoma cells (LA4 cell line) was used to study the possible mechanism of XQLT. Schematic of cell experimental groups is shown in Figure 1A. LA4 cells stimulated with Der p produced three times more NGF than un-stimulated cells did (“D” and “N” in Figure 1A). Cells with XQLT treatment alone (XC) exhibited decreased NGF expression compared to untreated cell (N). Treatment with XQLT alone inhibited the expression of NGF in LA4 cells without causing toxicity (by MTT assay, data not shown). Pre-treatment with XQLT (“XP” in Figure 1A) decreased NGF expression more than did co-treatment with XQLT (“XD” in Figure 1A). A single dose (determined in a pre-titration trial, whose results are not shown) of XQLT as a pre-treatment appeared to suffice for the inhibition Der p-induced NGF expression (“XP” in Figure 1A). LA4 cells exhibited high baseline levels of BDNF production. Der p stimulation slightly elevated LA4 BDNF levels, whereas XQLT clearly reduced them (“XP” and “XD” in Figure 1A). The levels of thymus-and activation-regulated cytokine (TARC), which is the cytokine that recruits eosinophil and Th2 inflammatory cells in the early phase of an allergic reaction, were also reduced in XQLT-treated LA4 cells (“XP” and “XD” in Figure 1A).

p75NTR knockout mice are known to have a lower response to allergic stimulation [20]. XQLT also inhibited the expression of p75NTR at the protein level in LA4 (“XP”, “XD” and “XC” in Figure 1B). Pre- and co-treatment (XP and XD) with XQLT indistinguishably reduce p75NTR levels. XQLT treatment (Figure 1B) also inhibited the expression of long-form pro-NGF, which was induced by Der p. A decrease in pro-NGF level might be responsible for the observed decrease in NGF level in the cell culture supernatant.

The article "Xiao-Qing-Long-Tang shows preventive effect of asthma in an allergic asthma mouse model through neurotrophin regulation" was published in 2013. Journal: BMC Complement Altern Med.

XQLT had a regulatory effect on neurotrophin and TARC from epithelial cells that were stimulated by Der p. An established acute asthmatic mouse model was then used to study how XQLT would affect neurotrophin in the asthma reaction.

### Measurements of respiratory flow resistance showed inhibition of AHR by XQLT in Der p-induced acute asthma

Figure 2A schematically depicts the experimental groups of mice. Figure 2B reveals that the Der p-challenged mice that had been preventively administered XQLT orally (Group P) had a significantly lower respiratory resistance than did the Der p-challenged mice that had not been treated with XQLT (Group D; p < 0.01 marked by * symbol). The preventive strategy also decreased the respiratory flow resistance significantly more than did the therapeutic strategy (Group T; p < 0.05 marked by # symbol). Mice treated with XQLT oral administration only (Group XC) had airway resistance similar to the airway resistance of naive mice (Group N). These results suggested that XQLT positively inhibited Der p-induced AHR in mice. The airway resistance of Group XC was not increased. Although XQLT has been found to inhibit AHR in Der p stimulated mice, the supported data was based on the indirect Penh method [3]. In this research, AHR values were measured directly via intubation in a mouse model of Der p-challenged acute asthma and could be more precise.

The article "Xiao-Qing-Long-Tang shows preventive effect of asthma in an allergic asthma mouse model through neurotrophin regulation" was published in 2013. Journal: BMC Complement Altern Med.

### BALF cytokine profile and eosinophil infiltration in the lung of the acute asthma mouse model

Both IL-5 and IL-13 are known to be involved in the recruitment of eosinophil. However, the data did not show that XQLT had any clear effect on IL-5 or IL-13 (Figure 3A). XQLT did not have any significant effects on IFN-γ levels in this Der p-induced acute asthma mice model (Figure 3A). However, the thymus-and activation-regulated cytokine (TARC), which is known to be involved in the Th2-cell attraction response and may be regulated by NGF [27], was greatly suppressed by both strategies of XQLT administration (Group P and Group T). If these relationships between NGF, BDNF and TARC were taken together, XQLT might regulate neurotrophin and TARC for showing preventive effect on asthmatic processes. To understand the possible pathways affected by XQLT, further research was conducted to find the target receptor of XQLT effect.

**Figure 3:** **BALF cytokine profile and eosinophil infiltration in the lung of a mouse model of acute asthma. (A)** BALF was collected for ELISA analysis to evaluate IL-5, IL-13, IFN-γ, TARC, and TGF-β1 levels. TARC levels were clearly decreased by XQLT (Group P and T). Values shown are the mean ± SD (Student’s t test versus Group D) of the six mice in each group. All experiments were repeated for at least three times. * means p < 0.05; *** means p < 0.01 **(B)** Eosinophil infiltration in the lungs of mice in acute asthma model. Lung sections were prepared for a special stain to identify eosinophil (light pink; as arrow pointed) and structure cells (deep blue). Eosinophil counts were calculated from 30 vision fields and listed at the bottom-left of the images in the bar plot. Values shown are the mean ± SD (Student’s t test versus Group D; * means p < 0.05; *** means p < 0.01) (n = 6 mice for each group). All experiments were repeated for at least three times.

The data obtained using specific eosinophil/mast cell staining kits revealed that Der p stimulation induced the infiltration of eosinophil (light pink cells; as arrow pointed in Figure 3B) into the lungs. Both preventive (Group P) and therapeutic strategies (Group T) reduced eosinophil infiltration (bottom-left bar graph in Figure 3B).

### Effects of XQLT on total and Der p-specific IgE, IgG1, and IgG2a levels in serum and BALF in Der p-induced acute asthma mice model

Monitoring immune-pharmacological and physiological effects is important when a decotion is used for study in an asthma animal model. Our analysis of Der p-induced antibodies revealed that XQLT (Group P and Group T) tended to decrease serum total IgE, IgG1, and IgG2a levels, particularly in mice that had been subject to preventive strategy (Figure 4A). Der p-specific IgE levels were not significantly altered by XQLT, but Der p-specific IgG1 and IgG2a levels were decreased by XQLT, especially in the preventive strategy group (Group P in Figure 4A). XQLT also reduced total cell infiltration in BALF (Group P and Group T in Figure 4B). Mice treated with XQLT alone (Group XC) had antibody quantities or cell infiltration similar to those in naïve mice (Group N). The results suggested that repeated XQLT treatments could decrease allergic inflammation in a mouse model of Der p-challenged acute asthma.

The article "Xiao-Qing-Long-Tang shows preventive effect of asthma in an allergic asthma mouse model through neurotrophin regulation" was published in 2013. Journal: BMC Complement Altern Med.

**Figure 4:** **Effects of XQLT on serum total and Der p-specific IgE, IgG1, and IgG2a levels in a mouse model of Der p-induced acute asthma. (A)** XQLT administration, especially as a preventive strategy, decreased serum total IgE, IgG1, and IgG2a levels. Der p-specific IgG1 and IgG2a levels were also decreased by the preventive XQLT strategy. * means p < 0.05; *** means p < 0.01 **(B)** Total cell infiltration in the lungs was also decreased by the action of XQLT. Values represent the means ± SD (n = 6 mice for each group, all experiments repeated for at least three times; * means p < 0.05; ** means P < 0.01; *** means p < 0.005). Student’s t test was performed versus Group D in **(A)** and **(B)**.

### XQLT inhibited NGF and BDNF levels in Der p-induced acute asthma

*Der p* stimulation evidently increased NGF levels in the serum and BALF (Figure 5A). The preventive strategy (Group P) clearly reduced NGF levels in BALF, whereas the effect of the therapeutic strategy (Group T) was uncertain (Figure 5A). Those results showed similar trends in compared with the trends of AHR measurements shown in Figure 2B. Our results suggested that XQLT might down-regulate the AHR response of asthma by regulating NGF, a factor in the early phase of asthma [28,29]. Serum NGF was not significantly affected in either the therapeutic or the preventive group (Figure 5A). The mechanism by which XQLT down-regulated NGF levels in the BALF without affecting serum NGF levels will be investigated further. The therapeutic strategy appeared not to cause significant differences of BALF NGF.

**Figure 5:** **XQLT decreased NGF and BDNF levels in a mouse model of acute asthma. (A)** NGF and **(B)** BDNF levels in the serum and BALF were measured after sacrificing the mice. Values shown are the mean ± SD (Student’s t test versus Group D) of the six mice in each group. The preventive XQLT strategy (P) decreased NGF and BDNF levels the most, particularly in the BALF and serum. * means p < 0.05; ** means P < 0.01; *** means p < 0.005.

The article "Xiao-Qing-Long-Tang shows preventive effect of asthma in an allergic asthma mouse model through neurotrophin regulation" was published in 2013. Journal: BMC Complement Altern Med.

In contrast, both the preventive and therapeutic strategies reduced BDNF levels in the serum more than in the BALF (Figure 5B). BDNF has been found to play a role in the late phase of asthma [14], and has been reported to be involved in the infiltration of eosinophils, which are known for their persistent activity in asthma, into the lungs [11].

### XQLT reduces Der p-induced p75NTR and TrkA expression in lungs

p75NTR knockout mice are known to have a lower response to allergic stimulation [20]. Immunofluorescence was shown as Total Area density in bar graph of Figure 6. Der p stimulation induced high level of p75NTR expression in the lung (Group D). Data herein revealed that XQLT reduced Der p-stimulated p75NTR in the lungs of acute asthmatic mice model. XQLT might affect the asthmatic reaction by regulating p75NTR expression (Figure 6A). The preventive and therapeutic oral strategies showed inhibitive effects of minor statistical difference on p75NTR, revealing that other inhibition mechanisms must exist (Group P and Group T in Figure 6A). The inhibition of p75NTR and BALF NGF by XQLT might together explain how XQLT prevents the Der p-induced asthmatic reaction. TrkA is also involved in NGF-related allergic reaction. Our data also showed that Der p-stimulated mice to which XQLT was orally administered expressed less TrkA in the lungs (Group P and Group T in Figure 6B) than did the Der p-stimulated mice (Group D).

**Figure 6:** **XQLT decreased Der p-induced p75NTR and TrkA expression in the lungs.** The Der p-challenged lung was used to be sliced for immunofluorescence staining with an anti-p75NTR antibody or an anti-TrkA antibody. **(A)** p75NTR **(B)** TrkA. The symbol {I} represented antibody isotype control. Fluorescence was measured by image analysis system and shown as total area density in the bar plot. Fluorescence area density was average fluorescence density values from 36-50 vision fields. Values shown are the mean ± SD (Student’s t test versus Group D) (n = 6 mice for each group). All experiments were repeated for at least three times. * mean p < 0.05; ** means p < 0.01.

## Discussion

XQLT has been reported to inhibit allergic reactions in mice models of both acute and chronic Der p-induced asthma [3,24]. In this study, the action of XQLT was found to inhibit allergic reactions which were correlated with the allergic asthma response. IgE levels (Figure 4A) and the extents of eosinophil and leukocyte infiltration (Figure 3B and Figure 4B) were reduced, causing the XQLT-induced down-regulation of any prolonged allergic reaction in the Der p-induced acute asthma model. Hence, in this mouse model, XQLT might affect the Th2 response, which is actively involved in allergic reactions. Yet IgG2a which is considered to be Th1 reaction product will be controversial because XQLT also decreased IgG2a. Der p induced more IgG1 than IgG2a that indeed indicated a Th2 favored reaction. It seemed that XQLT might also have an effect on Th1 reaction. By further analyzing cytokine such as IL-12 or IL-4 may reveal the nature of this controversy. Der p also induced obvious TGF-β1 which is known to induce Treg cell that inhibits T helper cell reaction including both Th1 and Th2 [30]. XQLT did not inhibit TGF-β1 (Figure 3A) in this research. Former research also indicated that XQLT induced CD4-CD8+ T cell or CD4-CD8- T cell [3] that usually represents phenotype of Treg cell. By analyzing IL-10 expression [31] and subset of infiltrated cell with different phenotype in BALF in the future will show how XQLT affect these factors thus regulating T helper reaction.

The article "Xiao-Qing-Long-Tang shows preventive effect of asthma in an allergic asthma mouse model through neurotrophin regulation" was published in 2013. Journal: BMC Complement Altern Med.

Yamada et al. [4] reported that XQLT treatment was effective in their mouse model of ovalbumin-induced acute asthma. After an ovalbumin challenge and the XQLT oral administration, elevated NGF level in the BALF has been observed [4]. Since NGF and other neurotrophin have been reported to be factors that are involved in asthmatic reactions, XQLT may influence allergic reactions in asthma by regulating neurotrophin.

In this study, a mouse model of Der p challenge-induced acute asthma was used to show that XQLT inhibited the release of NGF (Figure 5A) and p75NTR receptor expression (Figure 6A) in the lungs. The preventive XQLT strategy inhibited NGF expression more than the therapeutic XQLT strategy (Figure 5A). Therefore, XQLT down-regulated Th2 responses and inhibited allergic reactions. AHR, which can clearly indicate acute asthma attacks and is directly affected by NGF, was also reduced by XQLT (Figure 2B). The preventive XQLT strategy also inhibited the expression of p75NTR receptor more than did the therapeutic XQLT strategy. Although serial doses of XQLT were in the preventive strategy (Figure 5A), a single dose of XQLT in vitro, administered as a pre-treatment, was sufficient to inhibit Der p-induced NGF production (Figure 1A; XP). Pre-treatment of LA4 with XQLT (Figure 1A; XP) reduced both NGF and TARC levels, which finding was consistent with the *in vivo* data. Western blot assays revealed that pre-treating LA4 cells with XQLT inhibited p75NTR receptor and pro-NGF expression *in vitro* (Figure 1B). Hence, XQLT was predicted to have a preventive effect on the acute asthma.

The article "Xiao-Qing-Long-Tang shows preventive effect of asthma in an allergic asthma mouse model through neurotrophin regulation" was published in 2013. Journal: BMC Complement Altern Med.

Both *in vivo* and *in vitro* data revealed that XQLT clearly reduced BDNF levels. Pre-treatment with a single dose of XQLT *in vitro* reduced BDNF levels (Figure 1A; XP) more than did preventive XQLT administration *in vivo* (Figure 5B; Group P). BDNF has been reported to be a constitutive factor in the lungs and plays an important role in lung development [32]. The effects of BDNF are most apparent in the late phase of asthma, rather than in the acute phase [14], and BDNF has also been reported to affect the infiltration of eosinophils into the lungs [11]. BDNF also has an important role in smooth muscle hypertrophy which contributes to persistent late phase of asthma [15,33]. XQLT inhibited TARC (Figures 1A and 3A), which has been shown to be a factor that attracts eosinophil in early phase of immunological reactions [34-36]. XQLT also reduced BALF NGF (Figure 5A) which has been shown to be a survival factor of eosinophil in local compartments such as alveoli and bronchiole [11,13]. These results may elucidate the effects of XQLT on eosinophil, and help to explain how XQLT performs a prolonged regulatory function in latent asthma. XQLT targets both eosinophil and neurotrophin in allergic asthma, and this targeting is likely to support the preventive value of XQLT. By regulating BALF NGF, TARC and serum BDNF levels, XQLT may control allergic inflammation and eosinophil infiltration in both the early and the late phases of asthma.

The exact mechanisms of action of the components of XQLT decotion remain to be elucidated. By fractionation of XQLT with chromatographic methods, such as those involving silica gel columns, can further elucidate the mechanisms of XQLT, including the pharmacodynamics and interactions. This fractionation research of XQLT will enable treatment with XQLT to be more precisely monitored to increase the effectiveness of treatment of asthma patients. Nagai et al. [4] reported that XQLT treatment was effective in their ovalbumin-induced acute asthmatic mouse model and might provide a hint for studying the XQLT mechanism. In their research, one of the XQLT ingredients, Pinellaiae ternata, played an important role in decreasing OVA-specific IgE. Lee et al. [37] and Shin et al. [38] also provided data that Pinellaiae ternata might play a definite role in decreasing Th2 reaction in asthmatic animal models. Pinellaiae ternata is in highest proportion of XQLT components. It is worthy to know how Pinellaiae ternata will affect the neurotrophin in an asthma mouse model.

Our data revealed that XQLT influenced members of the neurotrophin family. According to internal medical principles and acupuncture practices in TCM, XQLT can be used to resolve symptoms or diseases that are associated with *qi* malfunctions of the bladder meridian, which used to be thought to be related to functions of the autonomic nervous system. By interfering with the neurotrophin, XQLT and its derivative decotions may act on the nervous system and thereby potentially regulate spinal or brain functions. Neurotrophin also appear to have a different role in the immune system, such as autoimmunity. One of our future goals is to extend the use of XQLT and its derivative decotions in the treatment of neurotrophin-related diseases of immune malfunction.

The article "Xiao-Qing-Long-Tang shows preventive effect of asthma in an allergic asthma mouse model through neurotrophin regulation" was published in 2013. Journal: BMC Complement Altern Med.

## Conclusion

In conclusion, XQLT regulates neurotrophin in a Der p stimulated cell line model and in an asthmatic mouse model. The effects of XQLT on neurotrophin may cause down-regulation of asthma reaction including AHR and eosinophil infiltration.

## Competing interests

The authors declare that they have no competing interests.

## Authors’ contributions

R-SC designed the study and performed the statistical analysis. S-DW and L-JL provided and discussed the animal model design, they also helped in surveying results of animal study. Y-CW helped statistical analysis and performed those techniques such as ELISA, western and cell culture. R-SC also participated in the sequence alignment and drafted the manuscript. S-TK and J-YW modified the design of study and sequence alignment of manuscript, they also made final approval to submit this manuscript. All authors read and approved the final manuscript.

## Pre-publication history

The pre-publication history for this paper can be accessed here:

http://www.biomedcentral.com/1472-6882/13/220/prepub
